The article "The expression of podoplanin protein is a diagnostic marker to distinguish the early infiltration of esophageal squamous cell carcinoma" was published in 2017. Journal: Oncotarget.

# The expression of podoplanin protein is a diagnostic marker to distinguish the early infiltration of esophageal squamous cell carcinoma

**DOI:** 10.18632/oncotarget.14596

**Published:** 2017-01-11

**Authors:** Guangyong Chen, Rui Xu, Bing Yue, Xue Mei, Peng Li, Xiaoge Zhou, Shoufang Huang, Liping Gong, Shutian Zhang

**Affiliations:** ^1^ Department of Pathology, Beijing Friendship Hospital, Capital Medical University, National Clinical Research Center for Digestive Diseases, Beijing, 10050 China; ^2^ Department of Gastroenterology and Hepatology, Beijing Friendship Hospital, Capital Medical University, National Clinical Research Center for Digestive Diseases, Beijing, 10050 China; ^3^ Department of Pathology, Basic Medical College, Capital Medical University, Beijing, 100069 China

**Keywords:** podoplanin, esophageal squamous cell carcinoma

## Abstract

The esophageal squamous cell carcinoma (ESCC) is usually develped from low-grade intraepithelial neoplasia (LGIEN) and high-grade intraepithelial neoplasia (HGIEN) to infiltrative squamous cell carcinoma. Till now, it remains hard to screen for infiltration at earlier stages, especially the differentiation between HGEIN and early infiltrative carcinoma. The purpose of this study is to determine a role of podoplanin in differentiating between HGEIN and early infiltrative squamous cell carcinoma. Totally 133 patients pathologically diagnosed with early ESCC and/or precancerous lesions were enrolled.The EnVision two-step IHC staining technique was applied using the monoclonal mouse anti-human Podoplanin antibody (clone number: D2-40). The expressions of PDPN protein on the basal layer of squamous epithelium lesions could be divided into three different patterns: complete type, incomplete (non-continuous) type, or missing type. A diagnosis of HGEIN can be made if the basal layer showed non-continuous or complete expression of PDPN and a diagnosis of early infiltration can be made if the expression of PDPN is completely missing. Our study confirmed that PDPN was a potential biomarker to identify the presence of early infiltrative squamous cell carcinoma.

## INTRODUCTION

The esophageal squamous cell carcinoma (ESCC) is usually develped from low-grade intraepithelial neoplasia (LGIEN) and high-grade intraepithelial neoplasia (HGIEN) to infiltrative squamous cell carcinoma [1]. Along with the progression of the disease, the squamous-cell nests of the precancerous lesions will unavoidably infiltrate into the lamina propria or even deeper sites. The infiltration of the advanced ESCC and early squamous-cell carcinoma is easily diagnosed if the teardrop-like, finger-like, or reticular infiltration is seen in the lamina propria. However, it remains hard to screen for infiltration at earlier stages, especially the differentiation between HGEIN and early infiltrative carcinoma.

According to the World Health Organization [2], ESCC arise from the hyperplasia of the neoplastic squamous epithelium, with its front end showing pushing edge, which is known as the “bulky outgrowth”. The hyperplasia can further progress into teardrop- and stripe-shaped infiltration and then infiltrative carcinoma. The bulky outgrowth is traditionally regarded as a carcinoma *in situ*. However, it remains unclear whether the bulky outgrowth means an early infiltration due to the lack of objective criteria [3]. Thus, new diagnostic markers are required for the diagnosis of the early infiltration. In the ESCC, it lacks a specific structure as the myoepithelial layer in breast cancer or the basal cell layer in prostate cancer. Podoplanin (PDPN) protein expression is always a sensitive and specific marker to display the lymphatic endothelial cells and identify any lymphatic invasion. While some authors [4–7] have also explored the potential correlation between its expression in squamous cell carcinoma and its lymphatic metastasis, we found that D2-40 was significantly expressed in the basal layer cells in the normal squamous epithelium but not in squamous cells above the basal layer. Therefore, in our current study, we tried to investigate the possibility of regarding this specific epithelial layer as a myoepithelial layer of the breast tissue and thus using it as an objective indicator for judging the infiltration.

## RESULTS

### Expression of PDPN in normal esophageal squamous epithelium (Figure 1)

To identify the expression of PDPN protein in esophageal squamous epithelium, we first detected the expression of PDPN protein in normal esophageal squamous epitheliums (*n* = 69) using IHC staining with specific anti-PDPN antibodies (Clone D2-40) and found that the expression of PDPN protein was specifically detected at the basal layer of squamous epithelium in the normal esophageal squamous epithelium, but not in other cellular layers of the epithelium. While the cell membranes were stained at different densities, the expression of PDPN protein was much stronger in the basal layer around the lamina propria papillae than in other layers in the epithelium. These results suggest that the expression of PDPN protein is a histological marker of the basal layer of esophageal squamous epithelium.

### The expression of PDPN protein positive basal cell layer in squamous precancerous lesions (Figures 2, 3)

The basal layer of the esophageal squamous precancerous lesions had two growth patterns: linear growth and bulky outgrowth of squamous epithelium. In the linear growth, the basal layer was flat bulky. In the outgrowth of squamous epithelium, the proliferated epithelial layer is squeezed downward the lamina propria and made it become bulky; meanwhile, the basal layer was wave-shaped.

As we demonstrated that the expression of PDPN protein is specifically detected in the basal layer of esophageal squamous epithelium (Figure 1), the expression of PDPN protein should be a marker to distinguish the early infiltration of esophageal squamous carcinoma. To test this hypothesis, we detected the expression of PDPN protein in different stages of squamous intraepithelial lesions.

**Figure 1:** The normal esophageal mucosa The squamous epithelium of the normal esophageal mucosa is flat, with its lamina propria papillae projecting into the epithelium (**A**) HE straining, low-magnification). The D2-40 is expressed in the cellular membrane of the basal layer of normal squamous epithelium; although the densities varied, its expression in the cellular membrane of the basal layer of squamous epithelium around lamina propria papillae is more prominent. The D2-40 also can clearly display the LECs in the lamina propria (EnVision method; (**B**, **C**, and **D**): low-magnification, high-magnification).

As shown in Table 1, we first detected the expression of PDPN positive basal cell layer in low-grade squamous intraepithelial lesions. Specifically, the complete PDPN positive expression was detected in 79 lesions (%) in the basal layer of normal squamous epithelium in samples with linear growth (*n* = 85) in all 93 LGD lesions. In all these positive samples, non-continuous PDPN + expression were detected in 6 lesions, suggesting that some diseased cells had became dominant in the basal layer. In 8 lesions showing bulky grow, the basal layer of normal squamous epithelium showed complete PDPN + expression. Interestingly, the expression of PDPN protein was not detective in the squamous epithelial cells outside the basal layers of any lesion.

**Table 1:** Changes of PDPN + basal layer in ESCC and precancerous lesions

		LGIEN (93 lesions)		HGIEN (174 lesions)		
Basallayer PDPNexpression pattern	Normal(69 lesions)	Bulky Outgrowth(8 lesions)	Linear Outgrowth(85 lesions)	Bulky Outgrowth(106 lesions)	Linear Outgrowth(68 lesions)	Infiltrative SCC(75 lesions)
Complete	69	8	79	48	59	6
Missing	0			27	2	61
Non-conplete	0		6	31	7	8

Next, we detected the expression of PDPN protein in the basal layer in HGEIN (Table 1). Among 174 HGEIN foci, linear growth was detected in 68 of them (%) and bulky growth was detected in 106 of them (%). More specifically, the basal layer of 59 HGEIN foci with linear growth showed complete PDPN positive expression. In 2 cases, the cell membrane of basal layer had none PDPN expression detected which indicate the basal layer missing. In 7 cases, the expression was non-continuous; in these cases the basal layer-deficit spaces were occupied by atypical tumor cells with poloidal disorder. Among 106 bulky HGIEN lesions, the expression pattern of PDPN had three types in the basal layer, including 48 lesions with complete expression; 27 lesions with missing expression and 31 lesions with non-continuous expression. In patients with missing expression, the poloidal disorder of cells in the basal layer, was replaced by atypical tumor cells. In lesions with non-continuous PDPN expression, the squamous epithelial layer was almost completely tumorized except a small number of residual basal layer cells were occasionally visible. In some lesions, PDPN protein was occasionally expressed in the cytoplasm or envelope of squamous epithelial cells outside of the basal layer.

### Histological changes of the basal cell layer in the infiltrative ESCC and its PDPN expression pattern (Figure 4)

A total of 75 infiltrative ESCC nests were found. The PDPN + basal cell layer around them had completely disappeared and replaced by dysplastic cells with different PDPN expression pattern. Furthermore, the expression of PDPN protein was not detected in the basolateral cells of 61 lesions. The PDPN expression showed non-continuous type in 8 lesions. Solid and cord-shaped arrangement was detected in 6 basal cell-like ESCC nests. The expression of PDPN protein was completed detected on cellular membrane in tumor cells. Scattered PDPN expressions were occasionally detected in cytoplasm or membrane in tumor cells outside the basolateral layer of cancer nests in some cases.

## DISCUSSION

In this study, we observed the changes of PDPN in the precancerous lesions of ESCC at different grades and in infiltrative ESCC.

### PDPN + basal layer cells in squamous epithelium may be a cell layer of special biological significance

Podoplanin (PDPN), a 38kDa mucin-type transmembrane glycoprotein, has been used as a specific marker for lymphatic endothelial cells. However, it can also be expressed in other tissues and cells such as in kidney podocytes, skeletal muscle, placenta, lung, heart, salivary glands, osteoblasts, mesothelial cells, and rat type I alveolar epithelial cells [8–11]. While its physiological functions remain unclear, PDPN may be involved in cell differentiation and development. Schacht et al found that PDPN was expressed, though in varying degrees, in the basal layer of squamous epithelium of the normal skin, cervix, and esophagus, suggesting that the basal layer cells have special immune phenotypes when compared with cells in other layers [12]. The PDPN + basal layer cells in the normal squamous epithelium may be cells in the special functional layer with specific biological and differentiation features [13].

As shown in our current study, normally D2-40 clone of PDPN was detected in the myoepithelial layer of the esophageal glands. In the cervix, it is specifically expressed in the basal layer of squamous epithelium of vagina and is partially expressed in the reserve cells in the glands and in the squamous metaplastic lesions in cervical glands. Thus, it may be a pluripotent stem cell that can be differentiated to either adenocytes or squamous cells. Thus, the PDPN positive basal cell layer, to certain degree, is similar to the cervical reserve cell layer and the mammary myoepithelial layer - both of them are functional layers with special morphologies and phenotypes that separate the epithelial and stromal layers. Naturally, we speculated that it might have a similar clinicopathological role in judging the infiltration of ESCC as it does for the infiltration of breast cancer.

### The missing type of PDPN expression in the basal cell layer is an objective marker of the early infiltration of ESCC

#### Changes of PDPN positive basal layer cells in ESCC and precancerous lesions

In our current study, the D2-40 clone of PDPN was used to specifically display the basal layer of esophageal squamous cells. In normal conditions, the basal layer was intact, and the cellular membrane was stained at varying intensities. In patients with LGEIN, the basal layer was intact and flat in most cases but could be missing in a few cases, although no obviously atypical tumor cell was found. In patients with HGEIN, bulky growth was found in most cases in which the basal layer could be intacted, or non-continuous, or completely missed.The basal layer may be progressed from intact to non-continuous and finally completely missed. In our current study, among the linearly distributed LGEIN and HGEIN, non-complete expression types of PDPN were seen in 9 cases and 5 cases, respectively, indicating that the intraepithelial infiltration of tumor cells may predict that the invasion of some ESCC may begin from the linear growth of tumor cells.

Among the infiltrative tumor lesions, some tumor cells showed PDPN - expression while others showed PDPN + expression; even among those with PDPN + expression, basal layers with complete PDPN expression around the cancer nests was still lacking. In our series, PDPN was completing expressed in 6 lesions showing basaloid ESCC, which may be explained by the differentiation of PDPN in different cell types during tumorigenesis.

### The expression status of PDPN in basal layer cells can be used as an objective marker of the early infiltration of ESCC

It has been speculated that the precancerous cells arises from the basal layer, which is composed of a layer of pluripotent stem cells, among which the diseased stem cells can be differentiated into PDPN + or PDPN – neoplastic cells [14]. The precancerous lesion is essentially the growth and development of neoplastic cells in the epithelial layer, during which the basal layer cells may still exist to varying degrees; in other words, the basal layer cells did not experience cancerous/invasive change and growth.

The basal layer remains intact when the low-grade tumors grow and develop in the epithelial layer; however, in patients with high-grade tumors, the atypical cancerous cells become more dominant and occupy almost the whole epithelial layer. Meanwhile, the normal basal layer cells are also occupied and destroyed and thus gradually disappear; only a small number of intrinsic basal cells remain, showing a non-continuous phenomenon. It can be regarded as a carcinoma *in situ* since there are still residual myoepithelial cells during the atypical ductal mammary hyperplasia. When the lesion further progresses, the tumor cells completely occupy the basal layer and the normal basal layer completely disappears. What does it mean?

In our opinion, when the esophageal HGEIN shows bulky outgrowth and the basal layer completely disappears, the tumor budding can have deep lamina propria invasion and is closer to the muscular layer of mucosa, showing an invasive growth trend. At that time the tumor cells dominate the epithelial layer and destroy the proper basal layer. This is the same case for breast cancer: after the cancerous hyperplasia of mammary ductal epithelium, its surrounding myoepithelial layer disappears; this condition should not be diagnosed as carcinoma *in situ*; rather, it should be judged as the earliest infiltrative carcinoma. The findings of our current study provided an objective standard for judging the conditions.

For esophageal squamous epithelium showing atypical bulky hyperplasia, whether it is an infiltrative lesion remains controversial. Similarly, another study based on electron microscopy also found that, after the atypical hyperplasia (bulky growth) of esophageal squamous epithelium, the pseudopods of many tumor cells had already broken through the basal membrane and entered the lamina propria, which was believed to be the earliest infiltration of tumor cells [15]. In our current study, the lamina propria under the bulky-growing cell nests was often accompanied by PDPN + fibroblast proliferation and lymphatic plasma cell infiltration/aggression, and other histological and cytological reactions, which were consistent with the interstitial reactive changes after early infiltration.

### Change of the basal layer of PDPN + squamous epithelial cells in esophageal cancer and precancerous lesions and diagnostic recommendations

During the routine biopsy, it is not difficult to identify esophageal LGEIN and HGEIN based on the tissue structures and cytological findings in routine HE sections. When HGEIN occurs, the lesion shows a bulky outgrowth and approaches the muscular layer of mucosa, which makes it more difficult to make a diagnosis of HGEIN or early infiltration. Our study confirmed that displaying the basal layer with D2-40 clone of PDPN is a potential biomarker to identify the presence of any infiltration. A diagnosis of HGEIN can be made if the basal layer showed non-continuous or complete expression and a diagnosis of early infiltration can be made if the expression is completely missing (Figure 5). Thus, this technique may be used as an objective indicator of early cancer infiltration. Thus, we proposed the algorithm that reflects the change of the basal layer of PDPN + squamous epithelial cells in esophageal cancer and precancerous lesions and the diagnostic recommendations (Table 2).

**Table 2:** Recommendations on the diagnosis of esophageal cancer and precancerous lesions basedon changes in PDPN+ basal layer

Traditional diagnosis	Recommended diagnosis	Histology		Immune phenotype
		Cytology	Basal structures	PDPN+ basal layer
LGEIN	LGEIN	Mild-moderate dysplasia,involving epithelial layer < 1/2	Linear outgrowthBulky outgrowth	Complete type
HGEIN	HGEIN	Severe dysplasia, involvingepithelial layer >1/2	Linear outgrowthBulky outgrowth	Complete typeNon-complete type
HGEIN	HGEIN with earlyinfiltration	Severe dysplasia,involvingepithelial layer >1/2	Linear outgrowthBulky outgrowth	Missing type

## MATERIALS AND METHODS

Totally 133 patients were enrolled in Department of Pathology, Beijing Friendship Hospital, Capital Medical University from October 2012 to January 2016. All subjects were pathologically diagnosed with early ESCC and/or precancerous lesions. All samples were fixed with 4% neutral formaldehyde solution for 16–48 hours and then embedded in paraffin and underwent Hematoxylin-Eosin (HE) and immunohistochemical (IHC) staining.

### Criteria for pathological interpretation

According to the WHO classification of tumours of the digestive system (2010 edition), these lesions were divided into LGIEN, HGIEN, and infiltrative squamous cell carcinoma.

### IHC staining method and interpretation criteria

The EnVision two-step IHC staining technique was applied using the monoclonal mouse anti-human Podoplanin antibody (clone number: D2-40) (Dako). Negative and positive controls were set for IHC staining, and the sections were developed with DAB.

With the lymphatic endothelial cells as the internal control, the expressions of protein PDPN in ESCC and precancerous cells as well as its expression in the basal layer of squamous epithelium were detected. The expressions of PDPN protein on the the basal layer of squamous epithelium is divided into three different patterns: complete type, incomplete (non-continuous) type, or missing type. The complete type is defined that the PDPN is completely displayed on the cell membrane of the basal layer of squamous epithelium, with intact single basal layer (Figure 2); the incomplete type (non-continuous) is defined that the expression of PDPN protein is detected on parts of the cell membrane of the basal layer of squamous epithelium, with relatively intact single basal layer, although non-continuous phenomenon does exist (Figure 3G); the lacking type is defined that the expression of PDPN protein is not detected at all on the cell membrane of the basal layer of squamous epithelium, and the basal layer completely disappears (Figure 3H). In our current study we mainly observed the changes of PDPN expression on the basal layer of squamous epithelium of ESCC and precancerous lesions (Figure 4).

**Figure 2:** Low-grade intraepithelial neoplasia (LGIEN) in esophageal mucosa The epithelial layer of the esophageal squamous mucosa is flat. Squamous cells in the basal layer of mucosa proliferate and become crowded. These cells have uniform shape and size, with thickened nuclear chromatin (**A**) HE staining, low-magnification). The D2-40 displayed its expression in the cellular membrane of squamous cells in IGIEN lamina propria papillae and among papillas; meanwhile, it clearly displayed the LECs in the lamina propria (**B**) EnVision method, low-magnification).

**Figure 3:** High-grade squamous intraepithelial lesions (HGEIN) and early infiltrative ESCC in esophageal mucosa Squamous epithelium in the center of esophageal squamous mucosa shows bulky outgrowth towards the lamina propria, and the basal layer of squamous epithelium shows a wave-like structure. The squamous cell nests have round and neat borders. The squamous cells in the basolateral tumor of mucosa proliferate and become crowded. The shape and size of these cells are uneven; poloidal disorder of cells is visible, along with thickened nuclear chromatin (HE staining; (A) low-magnification; (C) low-magnification); D2-40 displayed that it was completely expressed on the cellular membrane of tumor cells in the basal layer of the round HGEIN squamous epithelial nests; the expression was missing in some tumor cells in the basal layer of cell nests also showing bulky growth, although it showed non-continuous expression in the basal layer (EnVision method; (B) low-magnification; E, intermediate-magnification; (G) high-magnification). The squamous epithelial nests at the right side of mucosal tissue had irregular border. A small number of cells were detached from the squamous cell nests and infiltrated into the lamina propria. A diagnosis of early infiltrative well-differentiated ESCC was made. The D2-40 displayed that there was a completely missing pattern in tumor cells in the basal layer of the ESCC nests (HE staining; A: low magnification; (D) HE staining, low magnification). Meanwhile, the D2-40 antibody also clearly displayed the lymphatic endothelium in the lamina propria (EnVision method; G and H, high magnification), follicular dendritic cell (FDC) networks in the propria lymphoid follicles, and a small number of fibroblasts that had proliferated (EnVision method; B, low magnification).

**Figure 4:** Infiltrative ESCC of the esophagus After ESD resection, the infiltrative ESCC of esophagus invaded the submucosa (HE staining, (**A**) low magnification; (**B**) high magnification). The D2-40 displayed that the basolateral tumor cells in squamous cell cancer nests showed completely lacking expression pattern, whereas the basal layer of the squamous epithelium that had proliferated around it showed complete expression on the cellular membrane (EnVision method; (**C**) low magnification; (**D**) high magnification). The D2-40 displayed the FDC networks in lymphoid follicles that had proliferated around the cancer nests, the basal cell layer around the submucosal esophageal glands, and the fibroblasts that had proliferated around the cancer nests; in addition, PDPN expression was also detected in a small number of cancer cells in the cancer nests.

**Figure 5:** Change of the basal layer of PDPN + squamous epithelial cells in esophageal cancer and precancerous lesions and diagnostic recommendations Basal layer cells (brown cells) in esophageal squamous epithelium can be specifically displayed by the D2-40 as a special functional layer with the potential to differentiate into other cells. Along with the occurrence and progression of the precursor lesion (blue cells) of ESCC, the lesion showed linear hyperplasia in the basal layer (from bulky outgrowth to infiltrative growth). Accordingly, the basal layer changed from “complete” (**A**) to “non-continuous” (**B**) to “completely disappear” (**C** and **D**); the “non-continuous” and “missing” means the lesion is a high-grade intraepithelial neoplasia or even carcinoma *in situ*. A diagnosis of “early infiltrative carcinoma” should be made when the basal layer completely disappears. Thus, the D2-40 can effectively display the expression pattern of the basal layer and thus can be used as an objective marker of early infiltrative carcinoma. EP: epithelium; BCL: basal cell layer; MM: muscularis mucosae.

## References

[1] Wang GQ, Abnet CC, Shen Q, Lewin KJ, Sun XD, Roth MJ, Qiao YL, Mark SD, Dong ZW, Taylor PR, Dawsey SM (2005). Histological precursors of oesophageal squamous cell carcinoma: results from a 13 year prospective follow up study in a high risk population. Gut.

[2] Masayuki Imamura (2000). Superficial esophageal neoplasm: patholgy, diagnosis, and therapy.

[3] Bosman Fred T., Carneiro Fatima, Hruban Ralph H. (2010). WHO classification of tumours of the digestive system Lyon.

[4] Schlemper R, Dawsey S, Itabashi M, Iwata A, Kato Y, Koike M, Lewin K, Riddell R, Shimoda T, Sipponen P, Stolte M, Watanabe H (2000). Differences in diagnostic criteria for esophageal squamous cell carcinoma between Japanese and Western pathologists. Cancer.

[5] Chuang WY, Yeh CJ, Wu YC, Chao YK, Liu YH, Tseng CK, Chang HK, Liu HP, Hsueh C (2009). Tumor cell expression of podoplanin correlates with nodal metastasis in esophageal squamous cell carcinoma. Histol Histopathol.

[6] Yuan P, Temam S, El-Naggar A, Zhou X, Liu DD, Lee JJ, Mao L (2006). Overexpression of podoplanin in oral cancer and its association with poor clinical outcome. Cancer.

[7] Wicki A, Christofori G (2007). The potential role of podoplanin in tumour invasion. British Journal of Cancer.

[8] Dumoff KL, Chu CS, Harris EE, Holtz D, Xu X, Zhang PJ, Acs G (2006). Low podoplanin expression in pretreatment biopsy material predicts poor prognosis in advanced-stage squamous cell carcinoma of the uterine cervix treated by primary radiation. Mod Pathol.

[9] Breiteneder-Geleff S, Soleiman A, Kowalski H, Horvat R, Amann G, Kriehuber E, Diem K, Weninger W, Tschachler E, Alitalo K, Kerjaschki D (1999). Angiosarcomas express mixed endothelial phenotypes of blood and lymphatic apillaries: podoplanin as a specific marker for lymphatic endothelium. Am J Pathol.

[10] Kawaguchi H, El-Naggar AK, Papadimitrakopoulou V, Ren H, Fan YH, Feng L, Lee JJ, Kim E, Hong WK, Lippman SM, Mao L (2008). “Podoplanin: a novel marker for oral cancer risk in patients with oral premalignancy,”. Journal of Clinical Oncology.

[11] Patil Ashok, Patil Kishor (2015). Suyog Tupsakhare, Mahesh Gabhane, Shrikant Sonune, Shilpa Kandalgaonkar. Evaluation of Podoplanin in. Oral Leukoplakia and Oral Squamous Cell Carcinoma. Scientifica (Cairo).

[12] Wicki A, Lehembre F, Wick N, Hantusch B, Kerjaschki D, Christofori G (2006). Tumor invasion in the absence of epithelial–mesenchymal transition: podoplanin–mediated remodeling of the actin cytoskeleton. Cancer Cell.

[13] Schacht V, Dadras SS, Johnson LA, Jackson DG, Hong YK, Detmar M (2005). Up-regulation of the lymphatic marker podoplanin, a mucin-type transmembrane glycoprotein, in human squamous cell carcinomas and germ cell tumors. Am J Pathol.

[14] Martin-Villar E, Scholl FG, Gamallo C, Yurrita MM, Munoz-Guerra M, Cruces J, Quintanilla M (2005). Characterization of human PA2.26 antigen (T1alpha-2, podoplanin), a small membrane mucin induced in oral squamous cell carcinomas. Int J Cancer.

[15] Takubo Kaiyo (2008). Pathology of the Esophagus: An Atlas and Textbook.

